The article "Stearoyl-CoA Desaturase 1 Potentiates Hypoxic plus Nutrient-Deprived Pancreatic Cancer Cell Ferroptosis Resistance" was retracted in 2022. Reasons: duplicated images; unreliable data.

# Stearoyl-CoA Desaturase 1 Potentiates Hypoxic plus Nutrient-Deprived Pancreatic Cancer Cell Ferroptosis Resistance

**DOI:** 10.1155/2021/6629804

**Published:** 2021-04-01

**Authors:** Jie Gao, Zhengyang Zhang, Yanfang Liu, Zining Zhang, Ming Wang, Aihua Gong, Lin Xia, Xiang Liao, Dongqing Wang, Haitao Zhu

**Affiliations:** ^1^Department of Medical Imaging, The Affiliated Hospital of Jiangsu University, Zhenjiang, China 212001; ^2^School of Medicine, Jiangsu University, Zhenjiang, China 212013; ^3^International Genome Center, Jiangsu University, Zhenjiang, China 212013

## Abstract

Hypoxia and nutrient starvation (H/NS) microenvironment, a notable characteristic of pancreatic carcinoma, plays a critical role in cell death resistance and tumor recurrence. However, its role in ferroptosis remains to be classified. Here, we found that H/NS contributed to the pancreatic cancer cell ferroptosis resistance depending on the altered intracellular lipid compositions. Mechanistically, H/NS induced the upregulation of stearoyl-CoA desaturase 1 (SCD1), which promoted monounsaturated fatty acids (MUFAs) synthesis and protected against lipid peroxidation. Surprisingly, SCD1 showed a strong correlation with antiferroptosis gene expression. Moreover, short-hairpin RNA-based knockdown of SCD1 enhanced erastin-induced ferroptosis *in vitro* under H/NS. Finally, our results demonstrate the synergistic effect of erastin and A939572, a special SCD1 inhibitor, in dictating pancreatic carcinoma subcutaneous ferroptotic death. Taken together, our findings reveal a new role of the H/NS microenvironment against ferroptosis and suggest a potential therapeutic strategy for overcoming ferroptosis resistance in pancreatic cancer cells.

## 1. Introduction

Due to the imbalance of unlimited proliferation of cancer cells and poor supplement of blood vessels, hypoxia and nutrient starvation (H/NS) has been recognized as the most important characteristic of pancreatic carcinoma microenvironment [1, 2]. H/NS microenvironment is not only the driver of pancreatic cancer cell growth and metastasis but also inducing cancer cell death resistance, which ultimately results in therapy failure. Therefore, it is necessary to investigate the mechanisms underlying the H/NS microenvironment mediating the cancer cell death resistance.

Ferroptosis, a newly identified type of programmed cell death, is characterized by iron-dependent lipid peroxidation [3]. Recently, more and more researches demonstrated tumor microenvironment, and energy materials were also critical regulators of ferroptosis [4, 5]. However, the exact mechanisms were still unclear. Under H/NS, cancer cells mostly depended on metabolism reprogramming, such as elevated de novo synthesis of fatty acids (FAs), for the sake of thriving [6, 7]. Extensive researches show that ferroptosis was tightly related to the FA balance. Polyunsaturated fatty acids (PUFAs) promote free radical generation and lipid peroxide accumulation, which act as a trigger for ferroptosis [8, 9]. Monounsaturated fatty acids (MUFAs) block the lipid ROS accumulation on the plasma membrane and further induce the ferroptosis-resistant state [10]. Stearoyl-CoA desaturase 1 (SCD1), a critical regulator of de novo synthesis, catalyzes the desaturation of saturated fatty acids (SFAs) to MUFAs [11]. These findings suggested that SCD1 may be involved in H/NS microenvironment-induced ferroptotic cell death resistance in cancer cells.

The article "Stearoyl-CoA Desaturase 1 Potentiates Hypoxic plus Nutrient-Deprived Pancreatic Cancer Cell Ferroptosis Resistance" was retracted in 2022. Reasons: duplicated images; unreliable data.

To test this hypothesis, we show that pancreatic cancer cells under H/NS condition are associated with the upregulation of SCD1 expression and ferroptosis inducer resistance. Silencing of SCD1 in H/NS cultured pancreatic cancer cells enhanced erastin induced ferroptosis *in vitro* and *in vivo*, which suggests a potential ferroptosis-based therapeutic strategy for pancreatic cancer.

## 2. Materials and Methods

### 2.1. Cell Culture

Human pancreatic cancer cell lines (BXPC3, SW1990, PANC1, and Patu8988) and mice pancreatic cancer cell line Panc02 were obtained from the Cell Bank of the China Academy of Sciences (Shanghai, China). Cells were cultured in high glucose Dulbecco's modified Eagle medium (DMEM) with 10% fetal bovine serum (FBS; ExCell FSP500) and antibiotics (100 units/mL penicillin, 100 mg/mL streptomycin) at 37°C in an incubator with a humidified atmosphere of 5% CO_2_. Hypoxic (H) incubation was performed at 94% N_2_, 5% CO_2_, and 1% O_2_. Nutrient starvation (NS) condition was performed in DMEM with 2% FBS and antibiotics (100 units/mL penicillin, 100 mg/mL streptomycin). H/NS condition was performed in DMEM with 2% FBS and antibiotics (100 units/mL penicillin, 100 mg/mL streptomycin) at 94% N_2_, 5% CO_2_, and 1% O_2_ for the indicated time (6, 12, and 24 hours).

### 2.2. Reagents

Erastin (#HY-15763), (1S,3R)-RSL3 (RSL3; #HY-100218A), sulfasalazine (SAS, #HY-14655), oleic acid (OA; #HY-N1446), or ferrostatin-1(Fer-1; #HY-100579) were purchased from MedChemExpress (MCE, USA). BODIPY-C11 (#D2861) was obtained from Invitrogen. Propidium iodide (PI) was purchased from KeyGEN BioTECH.

### 2.3. Cell Viability Assay

Cell viability was measured using Cell Counting Kit-8 (CCK-8; Dojindo, #CK04). PANC1 and Patu8988 cells were seeded into 96-well plates overnight, then exposed to conditions, and treated with reagents as indicated at the indicated time (6, 12, and 24 hours). Subsequently, 10 *μ*L of the CCK-8 solution with 90 *μ*L DMEM was added to each well of the plate to replace the original medium, incubated for 1-4 h at 37°C, 5% CO_2_. Then, the absorbance (OD value) at wavelengths of 450 nm was measured with a microplate reader (Biotek, #Epoch2).

The article "Stearoyl-CoA Desaturase 1 Potentiates Hypoxic plus Nutrient-Deprived Pancreatic Cancer Cell Ferroptosis Resistance" was retracted in 2022. Reasons: duplicated images; unreliable data.

Cells were seeded in 12-well plates at appropriate cell density and incubated overnight at 37°C containing 5% CO_2_ and then exposed to conditions and treated with reagents as indicated. Cell death was analyzed by SYTOX green (Invitrogen) or PI staining (KeyGEN) with microscopy.

### 2.4. Lipid Peroxidation Assay

The relative MDA level in cells or tumor issues lysates was measured using a Lipid Peroxidation (MDA) Assay Kit (Abcam, ab118970), and the experiments were carried out as described previously [12]. Cells or tumor tissues were homogenized with lysis buffer and the MDA in samples reacts with thiobarbituric acid (TBA) to generate an MDA-TBA adduct which can be quantified colorimetrically (OD = 532 nm).

C11-BODIPY imaging assay was performed to evaluate lipid peroxidation in cells. Briefly, cells were collected and stained with 5 *μ*M of BODIPY-C11 dye and 5 *μ*g/ml of DAPI. Pictures were photographed with a fluorescent microscope (Nikon, Japan).

### 2.5. Western Blot

Cells were lysed on ice for 30 min and centrifuged at 12,000×g for 10 min at 4°C. Protein concentrations were quantified using the bicinchoninic acid (BCA) assay (Invitrogen, #23225). Western blot assay was performed as described previously [13]. Antibodies were as follows: anti-human GPX4 (Abcam, #ab41787, 1 : 1000), anti-human SCD1 (Abcam, #ab19862, 1 : 1000), anti-human ACSL4 (Proteintech, #22401-1-AP, 1 : 1000), anti-human FTH1 (CST, #4393, 1 : 1000), anti-human NRF2 (CST, #12721, 1 : 1000), and anti-human *β*-tubulin (Abcam, #ab6046, 1 : 1000). Secondary antibody (either anti-rabbit or anti-mouse) was purchased from Thermo Fisher Scientific (Invitrogen). The blots were analyzed using the software ImageJ (Version 1.80, NIH, USA).

### 2.6. Quantitative Real-Time Polymerase Chain Reaction Assay (qRT-PCR)

Total RNA was extracted using RNAiso Plus (Takara) according to the manufacturer's instructions. For mRNA analysis, cDNA was synthesized from 1 *μ*g total RNA using the RevertAid First-Strand cDNA Synthesis Kit (Thermo, #K1622). The experiment was performed for reverse transcription according to the manufacturer's instructions. Subsequently, SYBR Green-based real-time PCR was performed in triplicate using SYBR Green master mix (Vazyme) on a QuantStudio 3 real-time PCR machine (Invitrogen). For analysis, the threshold cycle (Ct) values for each gene were normalized to expression levels of ACTB. Analysis was performed using the QuantStudio Design and Analysis Software. The primers, which were synthesized and desalted from Genscript, are shown in Table 1.

The article "Stearoyl-CoA Desaturase 1 Potentiates Hypoxic plus Nutrient-Deprived Pancreatic Cancer Cell Ferroptosis Resistance" was retracted in 2022. Reasons: duplicated images; unreliable data.

### 2.7. RNAi and Gene Transfection

Cancer cells were seeded in 6-well plates to achieve a confluence of 40-50% overnight. To generate knockdown cells, cells were infected with lentivirus carrying shRNA followed by puromycin (1 *μ*g/ml) selection for 10-14 days. These established stable cell lines were maintained in DMEM containing 10% FBS and puromycin (0.75 *μ*g/ml) for further experiments. The specific shRNA sequences are listed in Table 2.

### 2.8. ELISA Assay

To measure the content of MUFAs, pancreatic cancer cells were seeded in 6 cm dishes to achieve a confluence of 40-50% overnight and then incubated in indicated conditions. Cells were collected and MUFA concentrations were measured using the Human MNSFA ELISA KIT (Fankewei, #F10525, Shanghai, China) according to the manufacturer's instructions.

### 2.9. Xenograft Tumor Models

Animal studies were approved by the Committee on the Use of Live Animals for Teaching and Research of Jiangsu University. Five-week-old female C57BL/6 mice were obtained from GemPharmatech Company and maintained under standard conditions in the Animal Center of Jiangsu University.

Panc02 cells (5 × 10^5^) were injected subcutaneously into the right dorsal flanks of C57BL/6 mice. When tumors reached a volume of 50-100 mm^3^, the mice were randomly divided into four groups (five mice per group) and treated with DMSO (control), erastin (20 mg/kg), A939572 (1 mg/kg), or erastin (20 mg/kg) + A939572 (1 mg/kg) every two days for two weeks. The tumor volume and growth speed were monitored every two days until the end point at day 14.

### 2.10. Patient Selection

To determine the expression of SCD1 in pancreatic cancer tissues and normal tissues, the datasets in GEO (GSE16515) concluding 52 samples were adopted. The Cancer Genome Atlas (TCGA) database (https://tcga.xenahubs.net/download/TCGA.PAAD.sampleMap/HiSeqV2.gz) including those from 183 pancreatic carcinoma patient specimens were utilized to further analyze the association of SCD1 expression level with overall survival and disease-free survival rate. High and low groups were defined as above and below the quartile, respectively.

### 2.11. Statistical Analysis

All data are presented as the mean ± standard error of the mean (SEM). Statistical analysis was performed using Prism 8 software. The differences between groups were analyzed using Student's *t*-tests, one-way analysis of variance (ANOVA), or two-way ANOVA. *P* < 0.05 was considered to reflect a statistically significant difference. All the experiments were repeated at least three times.

The article "Stearoyl-CoA Desaturase 1 Potentiates Hypoxic plus Nutrient-Deprived Pancreatic Cancer Cell Ferroptosis Resistance" was retracted in 2022. Reasons: duplicated images; unreliable data.

## 3. Results

### 3.1. Hypoxic and Nutrient-Deprived Condition Protects Pancreatic Cancer Cells from Ferroptosis

Hypoxia combination nutrient starvation (H/NS) is a notable characteristic of pancreatic carcinoma microenvironment and facilitates cancer cell death resistance. We firstly access the role of H/NS on pancreatic cancer cell ferroptosis. Ferroptosis inducer can be divided into system Xc^−^ inhibitors (such as erastin, sorafenib, or sulfasalazine) and GPX4 deletion or inactivation (such as RSL3). Erastin, sulfasalazine, and RSL3 could induce PANC1 and Patu8988 cancer cell death, which could be rescued by ferrostatin-1 (Fer-1), a ferroptosis inhibitor (Figure S1A). To mimic the H/NS condition, PANC1 and Patu8988 cancer cells were cultured with 2% FBS in a hypoxia chamber with 1% O_2_ and then treated with various ferroptosis inducers. Compared to normal culture condition (control), PANC1 and Patu8988 cancer cells cultured in H/NS condition were more resistant to the ferroptosis inducer for the indicated time (6 h, 12 h, and 24 h), which is similar to the presence of Fer-1 (Figures 1(a) and 1(b), Figure S1B and S1C). Due to GPX4 is a critical regulator of ferroptosis, we constructed a stable GPX4 knockdown PANC1 cell line (Figure S1D) and further evaluated the cell viability under normal and H/NS condition. Compared to parental cancer cells, the cell viability of GPX4-knockdown cancer cell was decreased under normal condition, while little change under H/NS condition (Figure 1(c)). Given that lipid peroxidation is one of the most crucial features in ferroptosis, we next evaluated intracellular malondialdehyde (MDA) levels, an end product of lipid peroxidation. Ferroptosis inducers (erastin, sulfasalazine, or RSL3) increased the MDA levels, which can be abolished under the H/NS condition (Figure 1(d)). The results indicated that H/NS condition rescued ferroptosis inducers or GPX4 depletion induced ferroptosis.

### 3.2. SCD1 Expression Is Positively Related to Pancreatic Cancer H/NS Condition and Progression

Monounsaturated fatty acids (MUFAs) could block the lipid ROS accumulation on the plasma membrane and induce a ferroptosis-resistant state in cells, especially in the hypoxia and H/NS condition [14, 15]. SCD1 is an endoplasmic reticulum enzyme that catalyzes the rate-limiting step in the formation of MUFAs. Therefore, we hypothesize that SCD1 is involved in H/NS condition rescued cancer cell ferroptosis. Kaplan–Meier analysis of the TCGA data showed a trend of that high SCD1 expression associated with low disease-free survival and overall survival rate (Figure 2(a)). Analysis of a gene expression database in Gene Expression Omnibus (GSE16515) indicated that SCD1 was upregulated in pancreatic cancer tissues compared with normal pancreatic tissues (Figure 2(b)).

The article "Stearoyl-CoA Desaturase 1 Potentiates Hypoxic plus Nutrient-Deprived Pancreatic Cancer Cell Ferroptosis Resistance" was retracted in 2022. Reasons: duplicated images; unreliable data.

To further explore the role of SCD1 in H/NS cultured pancreatic cancer cell ferroptosis, we firstly detected basal SCD1 expression under normal and H/NS conditions in PDAC cell lines Patu8988, PANC1, BXPC3, and SW1990, with relatively high SCD1 expression in PANC1 and Patu8988 cells, which were chosen for the further research (Figure 2(c)). Following cultured PANC1 and Patu8988 cells under H/NS condition for the indicated time, there was a significant upregulation of SCD1 in protein- and mRNA-expression levels (Figures 2(d)–2(e), Figure S1E). As the primary function of SCD1 is to regulate the production of MUFAs, we also tested the concentration of intracellular MUFAs in H/NS cultured cancer cells, and a higher concentration of MUFAs was observed (Figure 2(f)). Altogether, these findings suggested that SCD1 is closely correlated to the pancreatic carcinoma malignancy and H/NS microenvironment.

### 3.3. SCD1 Is a Suppressor of Ferroptotic Pancreatic Cancer Cell Death under H/NS

To further explore the role of SCD1 in H/NS involved pancreatic cancer cell ferroptosis, two stable knockdown cell clones (SCD1 shRNA1 and shRNA2) were established with high silencing efficiency verified by Western Blot and qRT-PCR (Figures 3(a) and 3(b)).

Compared to the control group, erastin could significantly induce the SCD1 knockdown pancreatic cancer cell death under H/NS condition (Figure 3(c)). Also, the cell viability of SCD1-knockdown cells under H/NS condition was decreased upon erastin treatment, which was reversed in the presence of oleic acid (OA) or Fer-1 (Figure 3(d)). Furthermore, knockdown of SCD1 significantly increased MDA production in H/NS cultured PANC1 and Patu8988 in the presence of erastin (Figure 3(e)). Given that MUFAs, products of SCD1-catalyzed reaction, negatively regulate ferroptosis, we therefore asked whether MUFA concentration was altered in SCD1 shRNA groups. ELISA assay results showed a marked decrease in MUFA concentration occurred in SCD1 shRNA groups under H/NS condition (Figure 3(f)).

TCGA database analysis also showed that SCD1 expression correlated with the expression of ferroptosis-resistant markers (ACSL3, SLC7A11, and NQO1) in pancreatic cancer (Figure 3(g)). Together, these results revealed that SCD1-mediated MUFA formation precipitates ferroptosis resistance under H/NS.

### 3.4. Inhibition of SCD1 Activity Sensitizes Pancreatic Cancer Ferroptosis *In Vitro* and *In Vivo*

Next, we test whether SCD1 inhibitor, A939572, may have a synergistic effect on inducing ferroptosis. As expected, pretreatment with A939572 productively sensitized pancreatic cancer cells to erastin induced cell death (Figures 4(a) and S2A), which could be rescued in the presence of Fer-1. Furthermore, MDA production and lipid ROS level were significantly increased under A939572 and erastin combination treatment, consistent with an increased feature of ferroptosis (Figures 4(b) and 4(c)). Moreover, the expression level of FTH1 and NRF2 increased, while no significantly changed of ACSL4 in cells treated with A939572 and erastin under H/NS (Figure S2B-F).

The article "Stearoyl-CoA Desaturase 1 Potentiates Hypoxic plus Nutrient-Deprived Pancreatic Cancer Cell Ferroptosis Resistance" was retracted in 2022. Reasons: duplicated images; unreliable data.

We next investigated whether A939572 and erastin have synergistic ferroptosis-inducing effect *in vivo*. Administration of A939572 and erastin reduced the size of Panc02 subcutaneous tumors in C57BL/6 mice by 26.5% and 35.6%, respectively, and the combination therapy further reduced the size by 80.3%, compared with vehicle-treated tumors at day 14 (Figures 4(d)–4(f)). Moreover, combination treatment of A939572 and erastin also significantly augmented MDA levels in tumor tissues (Figure 4(g)) and had little impact on GPX4 protein expression (Figure S2G). This data suggested that pharmacological inhibition of SCD1 enhanced ferroptosis in pancreatic cancer *in vitro* and *in vivo*.

## 4. Discussion

In the present study, we provided evidence that H/NS results in SCD1 high expression in PDAC cells. Furthermore, SCD1-mediated accumulation of MUFAs is involved in protecting PDAC cells from ferroptosis under H/NS condition. Importantly, combining ferroptosis inducers with SCD1 inhibitor showed a synergistic effect *in vitro* and *in vivo*.

As one of the most aggressive malignancy, PDAC therapy has no significantly breakthrough until now. The tumor microenvironment has been considered a crucial component of therapy resistance [16]. Hypoxia and nutrient deprivation are the two most striking features in the solid tumor microenvironment. Our results show that pancreatic cancer cells under H/NS condition were significantly resistant to the ferroptosis inducers, a novel form of tumor-suppressor function for cancer therapy. Cells adapt to the H/NS microenvironment depending on metabolism reprogramming [17]. Since hypoxia restrains glucose-based acetyl-CoA generation, cancer cells rely on glutamine or acetate as alternative substrates for acetyl-CoA generation to fuel their elevation of FA synthesis pathway [7, 18, 19]. Also, cancer cells mainly depend on the uptake of exogenous unsaturated FAs in the absence of oxygen [20, 21] and facilitate increased endogenous FA desaturation via upregulation of SCD1 expression in low-serum condition [22]. Expression of SCD1 and endogenous MUFA production increased under such H/NS condition according to our results. SCD1 plays a critical role in the de novo synthesis of FAs, catalyzing the conversion of saturated fatty acids (SFAs) into ∆9-monounsaturated fatty acids (MUFAs). Our data emphasized the essential role of SCD1 mediated MUFA production in such H/NS condition of PDAC, and this protective effect of SCD1 is consistent with the fact that blockade of SCD1 causes multiple changes in cellular lipid content and induces apoptosis and ferroptosis in ovarian cancer cells [15].

The article "Stearoyl-CoA Desaturase 1 Potentiates Hypoxic plus Nutrient-Deprived Pancreatic Cancer Cell Ferroptosis Resistance" was retracted in 2022. Reasons: duplicated images; unreliable data.

Lipid peroxidation is the driver of ferroptotic cell death. Acyl-CoA Synthetase Long-Chain Family Member 4 (ACSL4) induces cancer cell ferroptosis through promoting arachidonic acid (AA) and adrenic acid (AdA) peroxidation [23]. MUFAs did not upregulate GPX4 expression, which reduces reactive phospholipids hydroperoxides to unreactive phospholipid alcohol. However, MUFAs hinder the accumulation of lipid ROS on the plasma membrane and decrease PUFA incorporation into phospholipids [10]. Our study found that PDAC cells increase the production of MUFAs with upregulated SCD1 expression under H/NS condition, which provokes a ferroptosis-resistant cell state. Moreover, a potential PDAC treatment strategy was highlighted by combing ferroptosis inducers with SCD1 inhibitors to eliminate the resistant effect originating from TME.

Taken together, the current study reveals that the involvement of SCD1-mediated MUFA production results in a ferroptosis-resistant cell state under H/NS condition in PDAC cells (Figure 5). Further research is required to identify the novel PDAC therapy strategy in combination with SCD1 inhibitors and ferroptosis inducers.

## Figures and Tables

**Figure 1:** H/NS condition protects pancreatic cancer cells from ferroptosis. (a) PANC1 and Patu8988 cells were treated with erastin (5 *μ*M for PANC1 and 40 *μ*M for Patu8988), RSL3 (3 *μ*M for PANC1 or 5 *μ*M for Patu8988), or sulfasalazine (2 mM) cultured in normal or H/NS condition for 24 hours. Cell viability was measured using a CCK8 kit. (b) Representative images showing the induction of cell death in PANC1 cells treated with erastin (5 *μ*M), RSL3 (3 *μ*M), or sulfasalazine (2 mM) cultured under normal or H/NS condition with or without Fer-1 for 24 hours. (c) Cell viability was measured in Ctrl shRNA and GPX4 shRNA PANC1 cells cultured in normal or H/NS condition for 24 h. (d) PANC1 and Patu8988 cells were treated with DMSO (control), erastin (5 *μ*M for PANC1 and 40 *μ*M for Patu8988), RSL3 (3 *μ*M for PANC1 or 5 *μ*M for Patu8988), and sulfasalazine (2 mM) in normal or H/NS condition for 24 hours. The levels of MDA were assayed. SAS represents for sulfasalazine; RSL3 represents for (1S,3R)-RSL3; Fer-1 represents for ferrostatin-1; GPX4 represents for glutathione peroxidase 4; Nor represents for normal condition. H/NS represents for hypoxia combination with nutrient starvation condition. Experiments were repeated three times and the data are expressed as the mean ± SEM. ^∗^*P* < 0.05. ^∗∗^*P* < 0.01. ^∗∗∗^*P* < 0.001. ^∗∗∗∗^*P* < 0.0001.

The article "Stearoyl-CoA Desaturase 1 Potentiates Hypoxic plus Nutrient-Deprived Pancreatic Cancer Cell Ferroptosis Resistance" was retracted in 2022. Reasons: duplicated images; unreliable data.

**Figure 2:** SCD1 expression is positively related to pancreatic cancer H/NS condition and progression. (a) TCGA database analysis of the association of SCD1 expression with overall survival rate and disease-free survival rate of patients. (b) Expression of SCD1 in GEO database (GSE16515). Pancreatic tumor tissues compared to pancreatic normal tissues. (c) Basal SCD1 protein expression levels in Patu8988, PANC1, BXPC3, and SW1990 cells cultured in normal or H/NS condition were detected by western blot. *β*-Tubulin expression was detected as a loading control. (d, e) Western blot and qRT-PCR analysis of protein and mRNA expression levels of SCD1 in PANC1 and Patu8988 cells cultured in normal, nutrient starvation, hypoxia, or H/NS condition. *β*-Tubulin expression was detected as a loading control for western blot. ACTB mRNA expression was detected as a loading control for qRT-PCR. (f) ELISA-based analysis of the MUFA concentration in PANC1 and Patu8988 cells under normal and H/NS conditions. Nor represents normal condition. NS represents for nutrient starvation condition. Hy represents for hypoxia condition. H/NS represents for hypoxia combination with nutrient starvation condition. Experiments were repeated three times and the data are expressed as the mean ± SEM. ^∗^*P* < 0.05. ^∗∗^*P* < 0.01. ^∗∗∗^*P* < 0.001. ^∗∗∗∗^*P* < 0.0001.

**Figure 3:** SCD1-mediated MUFA formation protects PDAC cells from ferroptosis under H/NS. (a, b) Western blot and qRT-PCR analysis of shRNA-mediated knockdown of SCD1 protein and mRNA expression levels in PANC1 and Patu8988 cells. *β*-Tubulin expression was detected as a loading control. ACTB mRNA expression was detected as a loading control for qRT-PCR. (c) Sytox green staining analysis of PANC1 (Ctrl shRNA), SCD1 knockdown PANC1 (SCD1 shRNA1 and SCD1 shRNA2) cancer cells treated with erastin (5 *μ*M) under H/NS condition. (d) PANC1 (Ctrl shRNA), SCD1 knockdown PANC1 (SCD1 shRNA1 and SCD1 shRNA2), Patu8988 (Ctrl shRNA), and SCD1 knockdown Patu8988 (SCD1 shRNA1 and SCD1 shRNA2) cancer cells were treated with erastin (5 *μ*M for PANC1 and 40 *μ*M for Patu8988) with or without OA (80 *μ*M) and Fer-1 (1 *μ*M for PANC1 and 5 *μ*M for Patu8988) under H/NS condition. Cell viability was accessed via CCK8 assay. (e) MDA assay analysis of PANC1 (Ctrl shRNA), SCD1 knockdown PANC1 (SCD1 shRNA1 and SCD1 shRNA2), Patu8988 (Ctrl shRNA), and SCD1 knockdown Patu8988 (SCD1 shRNA1 and SCD1 shRNA2) treated with erastin (5 *μ*M for PANC1 and 40 *μ*M for Patu8988) with or without OA (80 *μ*M) under H/NS condition. (f) Human MNSFA ELISA Kit was used to detect the content of monounsaturated fatty acids (MUFAs) in PANC1 (Ctrl shRNA), SCD1 knockdown PANC1 (SCD1 shRNA1 and SCD1 shRNA2), Patu8988 (Ctrl shRNA), and SCD1 knockdown Patu8988 (SCD1 shRNA1 and SCD1 shRNA2) cancer cells under normal or H/NS condition. (f) Analysis of the TCGA database for the correlation SCD1 mRNA expression level with the ferroptosis (ACSL3, SLC7A11, NRF2, and NQO1). The results are presented by heat map: *n* = 183. OA represents for oleic acid. Fer-1 represents for ferrostatin-1. Experiments were repeated three times and the data are expressed as the mean ± SEM. ^∗^*P* < 0.05. ^∗∗^*P* < 0.01. ^∗∗∗^*P* < 0.001. ^∗∗∗∗^*P* < 0.0001.

The article "Stearoyl-CoA Desaturase 1 Potentiates Hypoxic plus Nutrient-Deprived Pancreatic Cancer Cell Ferroptosis Resistance" was retracted in 2022. Reasons: duplicated images; unreliable data.

**Figure 4:** Inhibition of SCD1 activity sensitized pancreatic cancer ferroptosis in vitro and in vivo. (a, b) PANC1 and Patu8988 cancer cells were pretreated with DMSO or A939572 (5 *μ*M) for 48 hours followed by the addition of erastin (5 *μ*M for PANC1 and 40 *μ*M for Patu8988) for an additional 24 hours. Cell viability was measured by a CCK8 kit (a). The relative levels of MDA were assayed (b). (c) Lipid ROS level was evaluated using fluorescent microscope images of BODIPY-C11 (oxidized, green; reduced, red). (d–f) C57BL/6 mice were injected subcutaneously with mice pancreatic cancer cells Panc02 (1 × 10^6^ cells/mouse) and treated with DMSO, erastin (20 mg/kg/i.p., every two days), A939572 (1 mg/kg/i.p., every two days), or erastin (20 mg/kg/i.p., every two days) + A939572 (1 mg/kg/i.p., every two days). (c) Tumor volume was calculated every two days. Representative photographs (d) and tumor mass (e) of isolated tumor tissues in each treatment group at day 14. (g) MDA levels in isolated tumors were assayed at day 14 after treatment. Experiments were repeated three times and the data are expressed as the mean ± SEM. ^∗^*P* < 0.05. ^∗∗^*P* < 0.01. ^∗∗∗^*P* < 0.001. ^∗∗∗∗^*P* < 0.0001.

**Figure 5:** Schematic representation of the mechanisms of SCD1 potentiating hypoxic plus nutrient-deprived pancreatic cancer cell ferroptosis resistance.

**Table 1:** Sequences of primers used for qRT-PCR.

Name	Direction	Sequence (5′-3′)
SCD1-human	Forward	CCTGGTTTCACTTGGAGCTGTG
	Reverse	TGTGGTGAAGTTGATGTGCCAGC
FTH1-human	Forward	TCCTACGTTTACCTGTCCATGT
	Reverse	GTTTGTGCAGTTCCAGTAGTGA
ACSL4-human	Forward	GCTATCTCCTCAGACACACCGA
	Reverse	AGGTGCTCCAACTCTGCCAGTA
NRF2-human	Forward	CACATCCAGTCAGAAACCAGTGG
	Reverse	GGAATGTCTGCGCCAAAAGCTG
GPX4-human	Forward	ACAAGAACGGCTGCGTGGTGAA
	Reverse	GCCACACACTTGTGGAGCTAGA
ACTB-human	Forward	CACCATTGGCAATGAGCGGTTC
	Reverse	AGGTCTTTGCGGATGTCCACGT

The article "Stearoyl-CoA Desaturase 1 Potentiates Hypoxic plus Nutrient-Deprived Pancreatic Cancer Cell Ferroptosis Resistance" was retracted in 2022. Reasons: duplicated images; unreliable data.

**Table 2:** Sequences of shRNAs.

Name	Sequence (5′-3′)
SCD1-shRNA1	CCGGCGTCCTTATGACAAGAACATTCTCGAGAATGTTCTTGTCATAAGGACGTTTTTG
SCD1-shRNA2	CCGGCTACGGCTCTTTCTGATCATTCTCGAGAATGATCAGAAAGAGCCGTAGTTTTTG
GPX4-shRNA	GATCGTGGATGAAGATCCAACCCAACTCGAGTTGGGTTGGATCTTCATCCAC TTTTTG

## Data Availability

To determine the expression of SCD1 in pancreatic cancer tissues and normal tissues, the datasets in GEO (GSE16515) concluding 52 samples were adopted. The Cancer Genome Atlas (TCGA) database(https://tcga.xenahubs.net/download/TCGA.PAAD.sampleMap/HiSeqV2.gz. sampleMap/HiSeqV2.gz) including those from 183 pancreatic carcinoma patient specimens were utilized to further analyze the association of SCD1 expression level with overall survival and disease-free survival rate. High and low groups were defined as above and below the quartile, respectively.

## Supplementary Materials

Supplementary Materials Figure S1: H/NS condition acts as a repressor of ferroptosis. Figure S2: A939572 enhances erastin-induced ferroptosis.
